# Design of Human Resource Management System Based on Deep Learning

**DOI:** 10.1155/2022/9122881

**Published:** 2022-07-20

**Authors:** Jinlong Li, Zhe Zhou

**Affiliations:** ^1^Department of Business Administration, Henan Finance University, Zhengzhou, Henan 450046, China; ^2^Department of Business Administration, Zhongnan University of Economics and Law, Wuhan, Hubei 430073, China

## Abstract

With the advent of the Internet era, the frequency and proportion of candidates obtaining recruitment information through the Internet is getting higher and higher, and the amount of human resources information such as talent information and postinformation has also increased unprecedentedly, which makes human resources services face the problem of information overload. At the same time, deep learning has achieved great success in a series of fields such as computer vision, natural language processing, and semantic recognition in recent years. However, there are few related works in the field of deep learning applied to human resource management system at present. Therefore, this paper studies and improves the recommendation algorithm based on deep learning and applies it to the field of human resources recommendation. In order to improve the traditional and single algorithm of the existing recommendation system, and improve the performance of the human resource management recommendation system.

## 1. Introduction

At present, the recommendation algorithm based on deep learning technology has been implemented from theoretical research to practical application. Both enterprises and research scholars have carried out application research on deep learning technology to improve the quality of recommendation results. RecSys, a recommendation algorithm research organization, officially established a recommendation algorithm research group based on deep learning in 2016. It will help to promote the research and development of deep learning technology in recommendation algorithms and more encourage the use of deep learning recommendation algorithms [1, 2]. Zheng et al. achieved score prediction optimization by combining a convolutional neural network and factorization machine model to alleviate the problem of data sparsity and enhance the predictability of the model [3]. Wu et al. generated textual comment information through the LSTM (Long Short-Term Memory) model that fused the latent states of users and items. It is used as an auxiliary task to improve the prediction of the score, thereby improving the accuracy of the score prediction. At the same time, the personalized recommendation ability of the model is enhanced by using textual comment and rating information [4]. It can be seen that the research combined with deep learning technology will become the trend of recommendation algorithm development. The research of recommendation algorithm based on deep learning has a certain practical research value.

At present, a small number of research results of the human resource management system at home and abroad are integrated. The limitations of traditional recommendation algorithms and the performance bottlenecks in recommendation system have always been the stumbling block to the development of the field of human resource recommendation. At the same time, it also hinders the development of enterprises engaged in Internet human resources recruitment in the industry and can not provide practical and reference value application cases for technological innovation of enterprises.

Based on the above-given research status, this paper studies and improves the recommendation algorithm based on deep learning and applies it in the field of the human resource management system (HRMS). It proves the application feasibility of recommendation algorithm based on deep learning in this field and improves the attention of academia and industry in this research direction. The research on the design of a human resource management system based on deep learning has certain practical significance.

## 2. Deep Learning Technology and Recommendation Algorithm

### 2.1. Deep Learning Technology

Deep learning is the technical core of the current artificial intelligence research boom and an indispensable tool in the era of artificial intelligence, which enables researchers to focus more on solving key macro problems. The neural network algorithm is one of the representative algorithms of deep learning, mainly including the Deep Belief Network (DBN), Recurrent Neural Network (RNN), and Convolutional Neural Network (CNN). This paper mainly introduces the neural network, convolutional neural network, and mainstream framework of deep learning in detail.

#### 2.1.1. Neural Networks

The neural network model is a collection of artificial neurons composed of perceptrons. It is inspired by neurons in biology and is a model used in the field of mathematics. The neuron structure is shown in Figure 1 [5]. The structure of the neural network model is a group of associated neuron combinations, which are connected with each other in an acyclic graph [6]. Neural network models are generally organized into different levels of neuron representation, usually including the input layer, hidden layer, and output layer.

With the deepening of the theoretical research foundation, neural network models have produced many different structural representations, such as recurrent neural networks suitable for feedback loops, automatic encoders with symmetric structures, and convolutional neural networks for obtaining high-dimensional feature representations. In the recommendation algorithm of the human resource management system designed in this paper, the convolutional neural network is used as the basic model of potential association learning and high-dimensional representation feature extraction.

#### 2.1.2. Convolutional Neural Network

A convolution neural network is a model belonging to the structure of the neural network. The main characteristic is to use the operation of convolution operation for model training [7]. A convolutional neural network takes the classification or regression task as the final output and formalizes the target task into an objective function. By calculating the error or loss between the predicted value and the real value, the convolutional neural network feeds back the error or loss from the last layer to the front layer by layer according to the back propagation algorithm. That is, through the feedback operation, the layer parameters are updated layer by layer, and feed forward again after the update is completed. The two operations are iterated alternately until the network model training converges to achieve the purpose of model training. The specific mathematical expressions are shown in formulas (1) and (2).

(1) $$\begin{array}{c} x^{1}⟶w^{1}⟶x^{2}⟶\cdots ⟶x^{L-1}⟶x^{L}⟶w^{L}⟶z. \end{array}$$

(2) $$\begin{array}{c} z=f\left(x^{L},y\right), \end{array}$$

where *x*^*L*^ is the data input of the *L* layer, *w*^*L*^ is the relevant weight of the *L* layer, *z* represents the loss function of this calculation process, *y* is the final real classification mark, and the function *f*(·) takes as *w*^*L*^ the calculation parameter.

#### 2.1.3. Deep Learning Framework

With the promotion of the upsurge of deep learning technology, the research in the field of deep learning has been deepened. At the same time, the development framework corresponding to deep learning has also been greatly developed. At present, many mainstream frameworks have been widely used. Researchers can more conveniently construct the model of deep learning, promote the research process of deep learning, and accelerate the development of the industrialization of applied research of deep learning technology.  Table 1 shows the comparison and introduction of the simple functions of several mainstream frameworks based on deep learning, such as Tensor Flow, Caffe2, Theano, and Keras.

The algorithm in this paper is based on the model construction implemented by the Keras open source framework. The Keras development interface documentation and other materials are relatively complete. It can be combined with Tensor Flow and Theano technologies as the back-end foundation and can use GPU for parallel operation. At the same time, the Keras framework also supports the expansion of the distributed operation, providing reliable technical support for the subsequent transformation of distributed operation of algorithms.

### 2.2. Algorithm Recommendation

The existing recommendation algorithms based on deep learning mostly adopt the algorithm combining the deep learning model with the traditional recommendation algorithm. The depth models used include Restricted Boltzmann machine (RBM) [8, 9], CNN [10], RNN [11], and Stacked Denoising Autoencoder (SDA) [12]. RBM and SDA are classical and effective in the fusion recommendation algorithm. This section will focus on them.

#### 2.2.1. Restricted Boltzmann Machine

A restricted Boltzmann machine (RBM) is a structural model with a full connection between layers and no connection within layers. Its structure is shown in Figure 2. Here, *v*_*i*_ (0≤*i* ≤ *m*) represents the visible node and constitutes the visible layer, and *h*_*j*_ (0 ≤ *j* ≤ *n*) represents the hidden node and constitutes the hidden layer. In RBM, the visible layer usually represents the original input data. The hidden layer represents the data generated through learning and expresses the hidden features of the original data.

#### 2.2.2. Stacked Denoising Autoencoder

The structure of an autoencoder is similar to that of a single hidden layer perceptron. Its working process includes two parts: encoding and decoding. The encoding stage maps the input data to the feature space, and the decoding stage maps the encoded data back to the original sample space [13]. Inspired by the deep neural network, the literature connects multiple autoencoders and builds a deep network in the form of a stack. Taking the features extracted by the previous layer of autoencoders as the original input of the latter layer of autoencoders, so that a stacked autoencoder model is formed [14]. Its structure is shown in Figure 3, where *x* is the input data, and *x*_recon_ and *y*_recon_ are the reconstructions of *x* and *y*, respectively.

The stacked denoising autoencoder model can realize the approximation of complex functions by using a multilayer nonlinear mapping structure. The model uses the “damaged” input to train the ability of each layer of the network to remove noise so that the encoder obtained by each layer of training has better fault-tolerant feature extraction ability. Therefore, the learned latent features also have better robustness.

### 2.3. Text Processing Technology

The existing recommendation system can better extract the structured feature information of users and projects and apply it in the recommendation algorithm as content information, but there are some obstacles in the utilization of unstructured data such as text and multimedia [15, 16]. For example, text information needs to be processed into structured feature vectors before it can be used in recommendation algorithms. Chinese text processing generally needs to go through two processes: Chinese word segmentation and text feature vectorization.

#### 2.3.1. NLPIR Chinese Word Segmentation

Chinese word segmentation refers to the process of dividing a Chinese text into words and recomposing word sequences according to certain rules. The words of English text are directly separated by spaces, while Chinese text can use punctuation marks to divide text units such as words, sentences, and paragraphs but cannot use symbols to directly divide words. Therefore, Chinese word segmentation is much more complicated and difficult than English. Chinese word segmentation is the premise of Chinese text information analysis [3, 17]. At present, some domestic scientific research institutions and research institutes have teams studying this technology and have also developed some open source projects of Chinese word segmentation, such as HTTP CWS, IK, paoding, nlpir, and Pangu word segmentation.

The Chinese word segmentation system NLPIR is a Chinese word segmentation tool developed by the Chinese Academy of Sciences. Since its birth in 2000, it has accumulated to 2014, and the number of users has reached 300,000. Based on the existing Chinese lexical analysis, it provides a complete semantic analysis function of the document, which can automatically extract information such as person names, place names, organization names, keywords, and abstracts from Chinese texts. It is an important tool for Chinese information processing [18].

#### 2.3.2. Text Feature Vectorization

After Chinese word segmentation divides the text into word sequences, it needs to be further converted into feature vectors. There are two commonly used methods of text feature vectorization: word frequency-inverse document frequency (TF-IDF) and count-based vectorization [2, 19].

TF-IDF is a feature vectorization method commonly used in text analysis processing, which can evaluate the importance of words in a document in a corpus [20, 21]. The main principle is that if a word occurs frequently in individual documents, but infrequently in other documents, the word will get a higher weight after being calculated by TF-IDF.

Another way to vectorize text features is to convert documents into a Bag of Words vector by counting. The Bag of Words vector model ignores factors such as the grammar and word order of the text and regards it as a collection of a certain number of words. The events of all words in the document are independent of each other.

## 3. Overall Design of Recommendation Algorithm

### 3.1. Algorithm Requirements

In the human resource management system, there are mainly two types of data: one is the data related to the applicant, including the applicant's personal basic information, educational experience, skills and expertise, work experience, interested job types, and treatment requirements. As well as the feedback information of candidates in the process of using the recommendation system. This category is collectively referred to as user data [22]. The other type is job-related data, including the type of job of the job, the information of the recruiting company, job content, salary, benefits, and basic requirements for candidates. This category is collectively referred to as project data. The tasks of the HRMS are based on the user and project data present in the system. The recommendation algorithm is used for calculation and analysis to select jobs that may be of interest to candidates from a large number of jobs and recommend them to the candidates.

In a real recruitment website, the system first asks candidates to fill in basic personal information, which generally has fixed options for selection and is formatted information. In addition, the system will also provide more information to fill in columns such as self-introduction, educational background, work experience, and self-evaluation. These information have no fixed options and are nonformatted text information [23]. In the more professional recruitment process, companies even pay more attention to the personalized resume provided by the applicant. On the other hand, when companies publish job requirements on recruitment websites, in addition to providing basic formatted information such as salary ranges, working hours, and benefits, they may also add text information such as job descriptions and recruitment conditions as supplements. The text information in the resume is more targeted and professional than the customized template in the recruitment system. Whether it is for candidates or enterprises, the text description method provides them with a more flexible and effective way to describe their own content characteristics, and text information is also richer than structured information.

However, text information is different from structured information. It needs to be processed into structured feature vectors before it can be used in recommendation algorithms. In particular, for Chinese text processing, since there is no formal delimiter for words, the utilization of Chinese text information also needs to go through two processes of Chinese word segmentation and text feature vectorization [11, 24]. In addition, only a small part of the key content information in the text information really determines the user's preference and evaluation of the project. This part of the information is sparsely distributed in the high-dimensional vector, which is easily overwhelmed by other noncritical dimension information.

Based on the above-given reasons, in view of the difficulty in extracting and utilizing text information features in the field of HRMS, deep learning is used to extract hidden features. The strategy of integrating deep learning models and traditional collaborative filtering algorithms seems to be more appropriate.

### 3.2. Overall Design of Algorithm

The main idea of the recommendation algorithm of HRMS based on deep learning is to use the deep learning model to represent and learn the text information. Thus, the key hidden features of low dimension are extracted and used in the traditional collaborative filtering algorithm [25].

The overall process scheme of the recommendation algorithm of HRMS based on deep learning is shown in Figure 4. The latent semantic matrices U and V are, respectively, the latent factor vector sets of all users and items obtained by probability matrix decomposition, which are used to construct the predicted scoring matrix.

The preliminary preparation of the recommended algorithm of HRMS includes data acquisition and data preprocessing. The data collection stage is responsible for collecting information about candidates and jobs from the human resources business system [26, 27]. The data preprocessing stage is responsible for cleaning, transforming and reducing the collected data, and storing it in the data warehouse. Data preprocessing involves repeated data patching, such as deleting redundant data according to certain rules and filling in missing data. It is not a one-step process, and the processing rules need to be continuously improved in the preprocessing [28].

After the data preparation is completed, the user item scoring matrix and item text feature vector are constructed as the input of the hybrid depth collaborative filtering algorithm. The former is converted from behavior record information representing user preferences into scores through certain rules, while the latter uses job description information to construct the text feature vector of the project.

The hybrid deep collaborative filtering algorithm includes two submodule algorithms, namely, the deep model algorithm and the content-based filtering algorithm. The main body of the deep model algorithm consists of a stack denoising autoencoder and a probability matrix decomposition. The former uses its feature extraction ability to extract low-dimensional implicit feature vectors from high-dimensional item text feature vectors as a probability matrix. The probability matrix decomposition module uses the low-dimensional feature vector of the item and the original rating matrix to learn to obtain the latent semantic vector of the user and the item.

## 4. HRMS Based on Deep Learning

### 4.1. Overall Requirements and Design Ideas

The goal of the HRMS is to improve the user experience of candidates in the process of finding suitable jobs on the employment platform. Its most basic task is to recommend jobs of interest to candidates so that the recommended jobs have a high degree of matching with the candidates, thereby increasing the probability of candidates successfully obtaining jobs [29, 30]. In order to achieve this goal, the system needs to provide channels for candidates to upload and publish their own information. It is a channel for companies to postjobs and an entrance for candidates to get personalized job recommendations.

In general, the overall requirements of HRMS are roughly as follows:

1. Candidates can register, upload, and publish their own recruitment information.
2. Enterprises can publish new recruitment requirements in the system. It can provide basic information and text description information of the position.
3. Candidates can browse the list of personalized recommended jobs in the system.
4. Candidates can click to browse, save, and apply for the job records that they are interested in.
5. Candidates can manage and followup on favorites and applied for jobs.

Most of the above-given requirements belong to the basic business requirements of the system. The most critical requirement is the function of obtaining personalized job recommendation in the system. The quality of the personalized recommendation list determines the candidate's satisfaction with the recommendation system. In this paper, the HDCF algorithm is used to realize the personalized recommendation of human resources [31]. The algorithm can better overcome the problems of data sparseness and cold start of projects in human resource data. Therefore, the recommendation effect is better than that of the traditional recommendation algorithm.

There is also a real-time problem in the recommendation results; that is, after one update and before the next update, newly registered users and newly released jobs cannot be updated to the recommendation results in time. In response to this problem, this paper adopts two strategies to solve this problem: (1) recommending the most popular and latest jobs in the system for newly registered users; (2) using a content filtering-based algorithm to online calculate the candidate's rank for the latest posted jobs Predict scores and update to the score matrix.

### 4.2. Overall System Structure

The overall architecture of the human resource recommendation system is shown in Figure 5. In this paper, the recommendation system is divided into three layers, namely, the application layer, the middle layer, and the storage layer [32]. The middle layer includes the data preprocessing layer and the recommendation calculation layer. The application layer, data preprocessing layer, and recommendation calculation layer are maintained by their respective subsystems, and the functions between the two layers are called through interfaces.

The application layer is developed with Java Web technology to provide the interaction between candidates and the recommendation system. It is mainly divided into two parts: basic business application and postrecommendation application. The basic business application of HR includes the functions of registering, logging in, browsing jobs, collecting, and applying for jobs. The position recommendation application includes personalized position recommendation and the latest popular position recommendation [33]. It is responsible for presenting the list of positions recommended by the system to users. For normal users, the system uses the results obtained by the recommendation computing layer to make recommendations. When the logged-in user is a newly registered applicant, the latest and most popular jobs are used for recommendation.

The data preprocessing layer is implemented by the open source ETL tool Kettle, and its responsibilities include the following three points:

1. *Data Collection*. Collect user behavior log records from the application layer.
2. *Build a Data Warehouse*. Clean and convert the human resource data stored in the business database, build a human resource data warehouse for HDCF algorithm processing, including cleaning and conversion of users and item tables, analysis and extraction of behavior data from log records, construction of scoring matrix, and construction of word bag vector set of items.
3. *Scheduled Incremental Updates*. Use the kettle tool to set regular tasks, regularly detect whether there are newly added candidates or position data in the business data table, and timely synchronize the updated data to the data warehouse. When a new postrelease is detected, a notice is sent to the recommendation calculation layer.

The recommendation calculation layer is the core of the human resources recommendation system, which mainly includes the following responsibilities:

1. *HDCF Model Training*. It is used to score the depth of the HDCF application model in the warehouse to provide users with personalized data.
2. *Online Update of the Predicted Scoring Matrix*. After receiving the notification from the data preprocessing layer, the content-based filtering algorithm is applied to the newly added postitems. Based on the basic attributes of the job, its predicted score is obtained and updated into the score matrix used to provide personalized recommendations.
3. *The Latest Popular Job Statistics*. Count the latest released and popular job sets and recommend them to newly registered candidates. The system calculates a priority weight for each job position and selects the position with a higher weight value to form a recommendation set [34].

The storage layer is the foundation of the recommendation system and consists of MySQL and Redis. MySQL is used to store all data in the recommendation system, including user basic data, job data, user behavior data, data warehouse for model training, and calculation results of the recommendation layer [35]. Redis is used as a cache database to cache data such as the prediction score matrix and the latest popular recommendation list.

### 4.3. System Processing Flow

The basic processing flow of HR recommendation system is shown in Figure 6. The figure shows a series of the workflow of HR recommendation system from data collection to providing recommendation results to users.

As can be seen from the data label in Figure 6, the basic workflow of the recommendation system includes the following five steps:

1. As shown in the data flow shown in label ①, the Java Web application provides the candidate with basic business functions and shows the user the work list recommended by the recommendation system to the user.
2. As shown in the data flow shown by labels ②∼③, the ETL server reads raw HR data from my SQL database, cleans, and transforms. Thus, the warehouse data for HDCF algorithm model training is obtained and saved in my SQL database.
3. As shown in the data flow shown by the labels ④∼⑤, it is recommended that the calculation server reads the warehouse data from the MySQL database and performs two parts of calculation work. One part is to perform offline model training, and the predicted score matrix is obtained for a personalized job recommendation. The other part is to calculate the weight of the latest popular jobs and get the recommended list of the latest popular jobs.
4. As shown in the data flow shown by the labels ⑥ ⟶ ④ ⟶ ⑤, the ETL server regularly checks whether there is any new candidate or position information added in the business data table and sends a notification to the recommendation calculation server in time. Having it updates the predicted scoring matrix and the latest top recommendation list will update the synchronized Redis and MySQL databases.
5. As shown in the data flow shown by the labels ⑦∼⑧, the system caches the corresponding business data from my SQL to the Redis database according to the request sent by the Java Web application. At this time, Redis caches business data and recommendation calculation results and can efficiently respond to requests from applications.

## 5. Conclusion

This paper mainly studies and improves the HR recommendation algorithm based on deep learning. It is applied to the field of HRMS to improve the traditional and single current situation of using algorithms in existing recommendation systems. With the help of deep learning feature extraction capability, this paper overcomes the main problems of traditional collaborative filtering algorithms such as data sparseness and cold start. An HDCF algorithm is proposed to further improve the quality of HR recommendation. Based on the main workflow of the recommender system, the overall architecture of the HRMS is designed, and a prototype system of HR recommendation based on deep learning is implemented. The system can better overcome the cold start problem and provide high real-time recommendation results.

## Figures and Tables

**Figure 1:** Neuron structure diagram.

**Figure 2:** Schematic diagram of RBM structure.

**Figure 3:** Schematic diagram of the stacked autoencoder model.

**Figure 4:** Overall design flow chart of the algorithm.

**Figure 5:** HRMS architecture diagram.

**Figure 6:** Work flow chart of HRMS.

**Table 1:** Comparison of deep learning frameworks.

Development framework	Implementation language	Development interface language	Document completeness	Execution efficiency
Caffe2	C++, Python	Python/MATLAB	Complete	High
Deeplearning4j	C++, Java	Java/Scala/Python	Complete	High
Keras	Python	Python/R	Complete	High
Tensor flow	C++, Python	Python/C++/Go/R	Generally	Medium
PyTorch	Python, C	Python	Complete	High
Theano	Python	Python	Generally	Medium

## Data Availability

The data used to support the study are included in the paper.
